The article "Prognostic indicators for poor outcomes in low back pain patients consulted in primary care" was published in 2020. Journal: PLoS One.

# Prognostic indicators for poor outcomes in low back pain patients consulted in primary care

**DOI:** 10.1371/journal.pone.0229265

**Published:** 2020-03-27

**Authors:** Eduardo B. Cruz, Helena Canhão, Rita Fernandes, Carmen Caeiro, Jaime C. Branco, Ana M. Rodrigues, Fernando Pimentel-Santos, Luís A. Gomes, Sofia Paiva, Isabel Pinto, Rubina Moniz, Carla Nunes

**Affiliations:** 1 Physiotherapy Department, Setúbal Polytechnic Institute, Setúbal, Portugal; 2 Comprehensive Health Research Center, CHRC, Lisbon, Portugal; 3 EpiDoC Unit, CEDOC, NOVA Medical School, Lisbon, Portugal; 4 ACES Arrábida, The Regional Health Administration of Lisbon and Tagus Valley, Lisbon and Tagus Valley, Portugal; 5 Research Center in Public Health, National School of Public Health, Lisbon, Portugal; Chinese Academy of Medical Sciences and Peking Union Medical College, CHINA

## Abstract

**Background:**

Non-specific low back pain (NSLBP) is the most prevalent musculoskeletal condition in western countries and is associated with persistent disability and high consumption of health care resources. NSLBP patients first seek primary health care services but the outcomes are often uncertain. This study aimed to examine the clinical course of the outcomes and to identify prognostic indicators for poor outcomes in NSLBP patients who consulted primary care.

**Methods:**

A prospective cohort study of 115 patients seeking treatment for NSLBP in primary care was conducted. Participants were consecutively recruited by their General Practitioners (GPs) and then assessed at baseline and 2 and 6 months later. Baseline assessment included socio-demographic and clinical data, psychosocial factors, pain, disability, and health related quality of life (HRQoL). Pain, disability, HRQoL and global perception of change were also assessed at 2 and 6-months’ follow-up. In addition, information regarding the GP’ practice was collected. Poor outcomes were determined according to the cut-off point used to define a persistent disabling condition and the minimal important change established for disability, pain and for global perception of change. The relationship between variables on baseline and poor outcomes was modulated through binary logistic regression analysis. The significance of associations was evaluated at **≤** 0.05 p-value with 95% confidence intervals (CI) and adjusted odds ratios (AOR).

**Results:**

110 (94.8%) and 104 (89.7%) participants completed the follow-up assessment at 2 and 6 months, respectively. The mean age (±SD) was 48.06 ± 11.41, with 53.9%, (N = 62) reporting an acute presentation of NSLBP. Six months after GP consultation, 53.8% (N = 56) of the participants reported a persistent disabling condition. An “LBP episode of less than 12 weeks” [AOR: 0.26; 95% CI (0.10, 0.65); AOR: 0.34; 95% CI (0.14, 0.81); AOR: 0.21; 95% CI (0.09, 0.53)],”maladaptive psychosocial factors” [AOR: 2.06; 95% CI (1.40, 3.04); AOR: 1.82; 95% CI (1.27, 2.59); AOR: 1.72; 95% CI (1.20, 2.47)] were significantly associated with poor outcomes on disability, pain and global perception of change, respectively. Besides these factors, being employed reduces the chances of poor outcomes on disability [AOR 0.31; 95% CI (0.11, 0.92)].

**Conclusions:**

A large proportion of LBP patients seeking primary health care reported poor outcomes 6 months after GP consultation. Patients who report chronic LBP, maladaptive psychosocial factors and are unemployed have a significant increase in the risk of poor outcome. These findings suggest the need of implementing effective models of care able to provide early screening and appropriate treatment to those at greatest risk of a poor outcome.

**Trial registration:**

Current Controlled Trials NCT04046874 (August 6, 2019). Retrospectively registered.

## Introduction

Non-specific low back pain (NSLBP) is one of the most common health problems in society and causes considerable disability, work absenteeism, and use of health services [1,2]. A systematic analysis for the Global Burden of Disease (GBD) reported that NSLBP stands out as the leading musculoskeletal disorder because of a combination of high prevalence and greater disability associated with this health state [2,3]. In Portugal, LBP is the most prevalent rheumatic and musculoskeletal disease affecting a large proportion of the population (26.4%) with significant costs for society and a large impact on disability, perceived health and quality of life for the individual [4].

In contrast with this burdensome scenario, episodes of acute NSLBP (pain of less than six weeks) have good prognosis. Findings of a prognostic systematic review and meta-analysis indicate that a marked reduction in mean pain and disability is expected in the first 6–8 weeks [5]. Beyond that time frame period, improvement slows and the probability of developing a persistent disabling back pain condition improves for approximately 40% of the patients [6]. Some of these patients will recover while others will develop a persistent severe LBP condition. The latter account for most of the social and health costs associated with this condition [7–11].

Probably due to the rapid improvement from an episode of LBP, a large proportion of people do not seek care. A review of ten population-based studies reported a pooled prevalence of care seeking of 58% [12], most commonly requested by women, individuals with poor general health, and with more disabling or more painful episodes [12,13]. These patients first seek primary health care services where the outcomes are often uncertain or differ widely between studies [14]. In studies focused on the course of pain, functional status, or mixed outcomes conducted in primary care settings, the proportion of patients with a poor outcome at 6 months ranged from 2% to 48% [14–17]. This wide range regarding the probability of achieving a poor outcome is possibly due to differences in study populations (acute/ sub-acute or chronic), the timeframe used for recruitment (e.g. first two weeks after the onset) and the criteria used to define a clinically important improvement or recovery [13]. However, and overall, these results suggest that for many LBP patients ongoing symptoms and residual disability may be common.

The inconsistent results found for the course of outcomes are extensible for prognostic indicators. A review of prognostic indicators concludes that the reporting of the strength of association was very inconsistent among the studies [6]. Indicators such as body mass index, age, symptom duration, distress, maladaptive pain behaviors, higher depressive symptoms, previous episodes of low back pain, higher intake pain intensity and functional disability, general health status and job satisfaction are often reported as important prognostic indicators for the development of persistent low back pain [6, 13, 17–25]. However, most of the prospective studies have been carried out on patients with recurrent acute and sub-acute LBP [14,15, 17, 21–23]. NSLBP patients seeking primary care for LBP treatment are a mixture of acute, sub-acute and chronic pain patients and few studies have explored the course of outcomes and prognostic indicators in mixed samples of LBP patients, in particular in patients who consult primary care.

Since most of the LBP patients first use primary health care services, and given the projected increases in such a burden as identified by the GBD study [26] are likely to add significantly to the primary care workload, the early identification of prognostic indicators for patients at risk for developing persistent and disabling symptoms might be crucial to identify which patients will most likely benefit from early intervention to decrease the likelihood of poor outcomes and prevent the development of a persistent and disabling LBP condition. The aims of this study were to examine the clinical course of pain, disability, health related quality of life and global perception of change, and to identify prognostic indicators for poor outcomes in patients seeking primary care for an episode of NSLBP of any duration.

## Materials and methods

A cohort of 115 patients seeking treatment for active symptoms of low back, with or without leg pain, of any duration, was consecutively recruited from 7 different primary care units in Portugal during a 7 months period (February to September 2018). Ethical approval was granted by the Ethics Committee of Regional Health Administration of Lisbon and Tagus valley (ARSLVT) (REF 3562/CES/2018). All the participants received oral and written information about the study and provided their written informed consent prior to participating. The study followed the STROBE guidelines for reporting observational studies [27,28].

All patients were referred for the study by their GP and screened for eligibility by a research assistant. GPs were encouraged to assess and treat their patients as usual and make all the referrals they think are appropriate for their patients. Potential participants were informed that participating in this study would not dictate the treatment they received for their LBP.

Participants were eligible if they were aged between 18 and 65 years, able to read and speak the Portuguese language and have a diagnosis of NSLBP (with or without leg pain and of any duration), defined as pain limited to the region between the lower margins of the 12th rib and the gluteal folds” [1, 29–31]. They were excluded if they have clinical signs of infection, tumor, osteoporosis, fracture, structural deformity, inflammatory disorder, radicular syndrome, or cauda equine syndrome, if they have severe depression or other psychiatric condition, if they are pregnant, or if they have undergone back surgery in the prior 6 months.

Immediately following the GP consultation, the research assistant assessed the enrolled participants at baseline and then at 2 and 6 months follow-up. This time periods were chosen given the marked improvement that is expected in the first 6 to 8 weeks following a new episode/ exacerbation of a prior condition of LBP and because little additional change has been shown to occur beyond 6 months [32].

Baseline assessment included a socio-demographic and clinical questionnaire, the Numeric Pain Rating Scale (NPRS), and the Portuguese versions of the Start Back Screening Tool (SBST), Roland Morris Disability Questionnaire (RMDQ), and the EuroQol five-dimension (EQ-5D, 3L). Following this baseline assessment, participants were contacted by telephone by the same research assistant at 2 and 6 months follow-ups and were reassessed with the NPRS, RMDQ-PT and the EQ-5D. A Global Perceived Effect Scale (GPES) to assess patient perception of change of their back condition was added in the follow-up reassessments. In addition, and to characterize the diagnostic procedures/ treatments received in these practices, information regarding the requested imaging tests, medication prescribed, sickness certificates and the referral to physiotherapy or to other medical specialities or services was collected from the participants’ health electronic records.

### Sample size

The sample size calculations were performed according to the general rule for dichotomous outcomes, which suggests that 10 events are required per each prognostic association tested [33]. In the present study, a total of 10 prognostic factors were included. Given the use of different poor outcome criteria an estimation of the poor outcome rate is difficult. Thus, the sample size estimation was based on the assumption of an expected 50% of probability of poor outcomes, at least 5 candidate variables on the multivariable analysis, and an estimated loss of follow-up of 15%. These assumptions generated a sample size of a minimum of 112 participants.

### Prognostic indicators

Potential prognostic indicators were identified via a literature search [6, 13, 17–25]. They included: age (in years), gender, working status (active/ not working), referred leg pain (yes/no), NSLBP pain medication (yes/ no), and current episode duration (acute/ sub-acute **<** 3 months; and chronic **≥** 3 months), maladaptive psychosocial factors, current pain intensity, disability and HRQoL.

The Keele Start Back Screening Tool (SBST) is a screening tool aimed to subgroup patients with regard to their risk of developing persistent LBP in primary care settings [34]. The psychosocial subscale score of the Portuguese version of the SBST (SBST-PT) was used to assess the presence of maladaptive psychosocial factors [34]. This subscale screens for modifiable predictors of persistent disabling back pain, including, fear avoidance, anxiety, pessimistic patient expectations, low mood and how much the patient is bothered by their pain, providing a psychosocial distress score [34].

Disability was measured with the Portuguese version of the RMDQ. The RMDQ consists of 24 items that assesses the functional status over the past 24 hours in patients with LBP [35]. Each answer can be scored “0” or “1”, thus leaving a range of scores from 0 to 24, with higher scores indicating higher disability. The RMDQ has shown good validity and test–retest reliability with reported intraclass correlation coefficients (ICC) of 0.8 or more [35–37].

Pain intensity was measured with a numerical pain rating scale (NPRS). Participants were asked to rate the intensity of their current pain on a scale of 0 (**“**no pain**”**) to 10 (**“**worst possible pain**”**) [38]. The NPRS has proven to be valid and reliable in patients with LBP pain [39,40].

Health Related Quality of Life (HRQoL) was measured with the Portuguese version of the EQ5D, 3L [41]. The index of the health status of the individual, which varies from a higher value of "1" (corresponding to the best possible health), and "0" (death) [41,42], was calculated to assesse HRQoL based on status in 5 dimensions: mobility, self-care, usual activities, pain discomfort and anxiety/depression, each with 3 levels of severity (0 = ‘no problem’, 1 = ‘moderate problem’, or 2 = ‘extreme problem). The weight applied to the severity states was based on the Portuguese valuation study of the EQ-5D,3L [43].

The overall perceived effect of treatment was measured with the GPES. GPES is a transition scale designed to assess the patients’ perception of change of their back condition [44,45]. The GPES ranged from -5 (“vastly worse”) to +5 (“completely recovered”). The Portuguese version of the GPES (GPES-PT) showed adequate test-retest reliability, validity and responsiveness [46]. A score of ≥3 has been proposed as the value that best discriminate between participants who have improved from participants who remained the same [46].

### Poor outcomes

Patient poor outcomes were determined at 2 and 6-months follow-ups, according to two different criteria. The primary outcome considered in this study was “persistent disabling low back pain” defined as the presence of a score of ≥7 on the RMDQ. This score was previously used to classify patients with a persisting and disability NSLBP condition [34]. Accordingly, participants in the 2 and/ or 6-months follow-ups that reported a RMDQ score **≥**7 were classified as having a persistent and disabling NSLBP condition. The secondary outcome criteria used to define a poor outcome status was the minimal important change (MIC) used to categorize patient’s improvement/ no improvement regarding disability, pain intensity and perception of overall change. Previous studies have established the MIC for the RMDQ and NPRS at a reduction of ≥30% from their baseline score [47], and a GPES score of ≥3 points at the follow-ups [46]. The 30% improvement on the RMDQ/ NPRS was calculated as follows: [(baseline RMDQ/ NPRS score- final RMDQ/ NPRS score)/(baseline RMDQ/ NPRS score)] X 100. For both classifications ‘‘no improvement” in this study was used to indicate ‘‘poor outcome.”

### Data analysis

All statistical analyses were carried out using the SPSS version 24.0 (SPSS Inc., Chicago, IL). Descriptive statistics were computed to summarize the participants' characteristics and the course of clinical outcomes: pain, disability, and HRQoL. Changes between baseline and follow-ups of disability, pain intensity, and HRQoL scores were first checked for normality (Kolmogorov- Smirnov test) and then analyzed using an ANOVA Friedman test (given the non-normality of the data). Pairwise comparisons were performed with a Bonferroni correction for multiple comparisons [48].

Poor outcome rates were determined from the percentage of those that met the no improvement criterion (poor outcomes) compared to those that meet the improvement criterion. Binary logistic regression models were constructed using baseline variables as potential prognostic factors for poor outcomes. In the bivariate analysis, variables with a significance level of less than 0.20 progressed to the next phase of modeling [49,50]. Separate multivariate models, using backward conditional elimination method, were then built for poor outcomes status (NPRS/RMDQ/ GRCS of less than MIC; RMDQ score of ≥7), at 2 and 6 months follow-up. Odds ratios (ORs) and corresponding 95% confidence intervals (CIs) were calculated for all variables in the bivariate and multivariate analysis. All variables remaining in the final model had an OR with a *p* value less than 0.05.

Lastly, the ability of the final model to discriminate between participants who remained the same/ worse from participants who have improved was calculated from the area under the receiver operating characteristic curve (AUC) using the different MICs and the persistent and disabling condition values as the external criterion. An AUC of 0.5 indicates no discrimination and 0.9, excellent discrimination [50].

## Results

Of the 119 NSLBP patients referred to the study, 115 completed the baseline assessment (Fig 1). Of the 115 enrolled NSLBP patients, 110 completed the 2 months follow-up (5 dropouts) and 104 the 6-month’s follow-up (6 drop outs). Reasons for withdrawal were exclusively related with the impossibility to contact the participants.

**Fig 1:** Study flowchart.

Table 1 details the baseline characteristics of these 115 patients. The mean age (±SD) was 48.06 ± 11.41, and they were predominantly female (56%) and employed (76.7%). Approximately half of the participants (53.4%) were acute presentations of NSLBP with a mean (±SD) disability score (RMDQ) of 12.6 (±5.9) and mean pain intensity score (NPRS) of 5.4 (±2.56).

**Table 1:** Baseline characteristics of study population (n = 115).

Variables, descriptive measures	Categories	Mean (SD) or Frequency
Age (years), mean ± SD^a^		48.06 (±11.41)
Gender, no (%)		
Male		50 (43.5%)
Female		65 (56.5%)
Work status, no (%)		
Active		89 (77.4%)
Not working		26 (22.6%)
Episode duration, no (%)		
Acute/ sub-acute (<3 months)		62 (53.9%)
Chronic (≥3 months)		53 (46.1%)
Referred leg pain, no (%)		
Yes		76 (66.1%)
No		39 (33.9%)
Pain medication (at the moment), no (%)		
Yes		66 (57.4%)
No		49 (42.6%)
SBST^b^ overall score, mean ± SD		5.4 (± 2.1)
SBST^b^ Psychosocial subscale (Q5-9), mean ± SD		2.8 (± 1.3)
Pain intensity (NPRS^c^ 0–10), mean ± SD		5.4 (± 2.6)
Disability (RMDQ^d^ 0–24), mean ± SD		12.6 (± 5.9)
HRQoL^e^ (EQ5D,3L^f^ Index), mean ± SD		0.44 (± 0.23)

Values are numbers (percentages) unless stated otherwise.

^a^ Standard deviation

^b^ Start Back Screening Tool

^c^ Numeric Pain Rating Scale

^d^ Roland Morris Disability Questionnaire

^e^ Health Related Quality of Life

^f^ EuroQuol 5D, 3L.

### Primary care management

In terms of the diagnostic management strategies used by GP, 56.9% of the participants were referred for imaging tests (35.7% plain x-rays and 14.8% computerized tomography) and 4.6% for other medical specialities consultations. Medication was the main treatment strategy used (83.5%), with an average of two medications prescribed per person. Nonsteroidal anti-inflammatory drugs (NSAIDs) (81.4%) and muscle relaxants (60.8%) followed by weak opioids (19.6%) were the types of medication most often chosen by the GPs. Only 8.3% of patients having been referred for physiotherapy and 32.6% of the employed participants received a sickness certificate.

### Course of outcomes

On average and comparing to baseline data, disability score (RMDQ) improved by 3.4 points at 2 months and by 4.2 points at 6 months. Pain intensity score improved by 1.5 points at 2 months and by 2.1 points at 6 months, and HRQoL index scores improved by 0.17 and 0.12 points, at 2 and 6-month follow-ups, respectively (Table 2). The results of the Friedman test shown statistically significant improvements in the course of disability (χ^2^(2) = 25.164, *p*< 0.005), pain intensity (χ^2^(2) = 25.099, *p*< 0.005), and HRQoL (χ^2^(2) = 27.638, *p*≤ 0.005) during the 6-month period. Post hoc analysis revealed statistically significant differences in the 3 outcomes from baseline to 2-month follow-up and from baseline to 6-month follow-up, but not from 2 months and 6-month follow-ups (Table 2).

**Table 2:** Course of outcome scores of the NSLBP patients.

Self-reported Measures/ Outcome Criteria	Baseline (n = 115)	2 Months (n = 110)	*p*	6 Months (n = 104)	*p*
Disability (RMDQ ^1^ 0–24) (median)	13	8	< 0.005	8	< 0.005
Pain intensity (NPRS ^2^ 0–10) (median)	6	4	< 0.005	3	< 0.005
HRQoL (EQ5D ^3^ Index) (median)	0.45	0.59	< 0.005	0.59	< 0.005

^1^ RMDQ-Roland Morris Disability Questionnaire

^2^ NPRS- Numeric Pain Rating Scale

^3^ EQ5D- EuroQuol 5D, 3L.

Despite statistical significant improvements at 2 months follow-up, approximately half of the patients did not reach the established recovery criteria for disability and pain (50.9% in disability and 50% in pain intensity), and 47.3% of the participants did not perceived any change in their condition or feel the same or worse (Table 3). At the 6 months follow-up the percentage of participants with poor outcomes decreased to 42.3% for pain, but remained nearly constant for disability (49%) and for perception of overall improvement regarding patient´s back condition (46.2%). Six months after GP appointment 53.8% of the participants reported RMDQ scores compatible with persistent disability (RMDQ ≥ 7) (Table 3).

**Table 3:** Proportion of patients with poor outcomes according to the different criteria used.

Self-reported Measures/ Outcome Criteria	2 Months (n = 110)	6 Months (n = 104)
Participants with RMDQ^1^ ≥7	64 (58.2%)	56 (53.8%)
Participants with poor outcome on disability (improvement of < 30% RMDQ)	56 (50.9%)	51 (49%)
Participants with poor outcome on pain intensity (improvement of < 30% NPRS ^2^)	55 (50%)	44 (42.3%)
Participants not perceived a meaningful change in their condition (score of < 3 GPES^3^)	52 (47.3%)	48 (46.2%)

Values are numbers (percentages)

^1^ RMDQ- Roland Morris Disability Questionnaire

^2^ NPRS- Numeric Pain Rating Scale

^3^ GPES- Global Perceived Effect Scale.

### Prognostic factors

Tables 4 and 5 presents the results of the multiple logistic regression analyses for poor outcomes at 2 and 6 months after the initial GP consultation. Overall, pain duration and the presence of maladaptive psychosocial factors were the two independent baseline predictors consistently associated with poor outcome at 2 and 6 months.

**Table 4:** ORs (95% Confidence Intervals) for the associations between prognostic indicators and poor outcome status at 2 Months follow-up (n = 110).

Prognostic indicators	RMDQ^1^ ≥7 N = 64		MIC^2^-RMDQ <30% N = 56		MIC-NPRS^3^ <30% N = 55		MIC-GPES^4^ ≥3 N = 52	
	Unadjusted	Adjusted	Unadjusted	Adjusted	Unadjusted	Adjusted	Unadjusted	Adjusted
**Sociodemographic variables**								
Age (yr) continuous	1.0 (0.97–1.04)		1.03 (0.99–1.06)*		1.03 (0.99–1.07)*		1.0 (0.97–1.03)	
Gender (ref female)	0.85 (0.39–1.82)		0.70 (0.33–1.48)		0.54 (0.25–1.15)*		0.68 (0.32–1.44)	
Work status (ref not working)	0.73 (0.29–1.84)		0.50 (0.20–1.26)*		0.31 (0.12–0.81)**	0.31 (0.11–0.86)**	0.78 (0.32–1.91)	
**NSLBP characteristics**								
Duration of LBP episode (ref > 3 months)	0.60 (0.28–1.30)*	0.16 (0.05–0.51)**	0.30 (0.14–0.65)**	0.25 (0.10–0.58)***	0.34 (0.16–0.74)**	0.36 (0.16–0.82)**	0.36 (0.28–1.52)*	0.29 (0.13–0.67)**
Radiating leg pain (ref no)	2.52 (1.12–5.67)		1.6 (0.72–3.53)		2.16 (0.96–4.84)**		2.12 (0.94–4.80)	
LBP Pain medication (ref no)	1.15 (0.54–2.47)		0.51 (0.24–1.09)		1.15 (0.41–3.24)		0.76 (0.27–2.18)	
**Self-reported Measures**								
Psychosocial factors (SBST^5^ Psychosocial sub-score, 0–5)	1.43 (1.53–3.27) ***	1.77 (1.11–2.82)**	1.48 (1.09–2.02)**	1.73 (1.22–2.45)**	1.21 (0.90–1.62)		1.61 (1.17–2.21)**	1.72 (1.23–2.40)**
Pain intensity (NPRS 0–10)	2.24 (1.19–1.71)***		1.08 (0.93–1.25)		0.85 (0.73–0.99)**	0.84 (0.72–0.99)**	1.02 (0.88–1.18)	
Disability (RMDQ, 0–24)	1.24 (1.14–1.35)***		1.01 (0.95–1.08)		0.99 (0.93–1.05)		1.0 (0.95–1.07)	
HRQoL (EQ5D^6^ Index, 0–1)	0.05 (0.01–0.59)***		0.95 (0.18–4.09)		4.19 (0.53–33.2)*		0.66 (0.9–4.92)	
Area Under de Curve (AUC)		0.86 (0.79–0.93)		0.72 (0.63–0.82)		0.73 (0.63–0.82)		0.73 (0.64–0.83)

*P<0.2

**P<0.05

***P<0.01.

^1^ RMDQ- Roland Morris Disability Questionnaire

^2^MIC—minimal important change

^3^ NPRS- Numeric Pain Rating Scale

^4^ GPES- Global Perceived Effect Scale

^5^ SBST–Start Back Screening Tool

^6^ EQ5D- EuroQuol 5D, 3L

**Table 5:** ORs (95% Confidence Intervals) for the associations between prognostic indicators and poor outcome status at 6 Months follow-up (n = 104).

Prognostic indicators	RMDQ^1^ ≥7 N = 56		MIC^2^-RMDQ <30% N = 51		MIC-NPRS^3^ <30% N = 44		MIC-GPES^4^ N = 48	
	Unadjusted	Adjusted	Unadjusted	Adjusted	Unadjusted	Adjusted	Unadjusted	Adjusted
**Sociodemographic variables**								
Age (yr) continuous	1.03 (1.0–1.07)*		1.04 (1.01–1.08)**		1.04 (1.0–1.08)*		1.03 (1.0–1.07)*	
Gender (ref female)	0.78 (0.35–1.65)		0.48 (0.22–1.07)*		0.48 (0.22–1.08)		0.51 (0.23–1.13)*	
Work status (ref not working)	0.46 (0.18–1.19)*	0.30 (0.09–0.98)**	0.35 (0.14–0.92)**	0.31 (0.11–0.92)**	0.31 (0.12–0.81)*		0.38 (0.15–0.97)**	
**NSLBP characteristics**								
Duration of LBP episode (ref > 3 months)	0.58 (0.26–1.26)*	0.29 (0.10–0.83)**	0.33 (0.15–0.74)***	0.26 (0.10–0.65)***	0.42 (0.19–0.93)**	0.34 (0.14–0.81)**	0.26 (0.11–0.58)***	0.21 (0.09–0.53)***
Radiating leg pain (ref no)	4.45 (1.87–10.6)***		1.88 (0.82–4.27)*		1.48 (0.65–3.40)		1.88 (0.82–4.30)*	
LBP Pain medication (ref no)	1.67 (0.76–3.65)		1.01 (0.47–2.2)		0.73 (0.33–1.60)		0.70 (0.32–1.53)	
**Self-reported Measures**								
Psychosocial factors (SBST^5^ Psychosocial sub-score, 0–5)	2.24 (1.52–3.31)***	1.94 (1.23–3.06)***	1.79 (1.27–2.53)***	2.06 (1.40–3.04)***	1.72 (1.22–2.42)**	1.82 (1.27–2.59)***	1.52 (1.1–2.1)**	1.72 (1.20–2.47)**
Pain intensity (NPRS, 0–10)	1.26 (1.07–1.49)**		1.09 (0.94–1.27)		1.22 (1.03–1.43)**		1.12 (1.02–1.41)**	
Disability (RMDQ, 0–24)	1.17 (1.08–1.26)***	1.16 (1.05–1.28)***	0.99 (0.93–1.05)		1.02 (0.95–1.09)		1.0 (0.93–1.07)	
HRQoL (EQ5D^6^ Index, 0–1)	0.10 (0.01–0.64)**		0.56 (0.29–8.35)		0.64 (0.12–3.49)		2.52 (0.45–14.0)	
Area Under de Curve (AUC)		0.83 (0.75–0.91)		0.78 (0.69–0.87)		0.73 (0.63–0.83)		0.77 (0.68–0.86)

*P<0.2

**P<0.05

***P<0.01.

^1^ RMDQ- Roland Morris Disability Questionnaire

^2^MIC—minimal important change

^3^ NPRS- Numeric Pain Rating Scale

^4^ GPES- Global Perceived Effect Scale

^5^ SBST–Start Back Screening Tool

^6^ EQ5D- EuroQuol 5D, 3L

Persistent disabling symptoms at 2 and 6 months (RMDQ score of ≥7) were predominantly associated with the duration of the LBP episode and the presence of maladaptive psychosocial factors. Participants with a LBP episode of less than 3 months had a reduced OR for persistence of symptoms at 2 and 6 months, respectively (OR 0.16 95%CI 0.05 to 0.51, *p*≤0.05; OR 0.29 95%CI 0.10 to 0.83, *p*≤0.05). In contraire, high scores at the baseline on the SBST psychosocial sub score improve the chance of developing a persistent pain and disability condition (OR 1.77 95% CI 1.11 to 2.82, *p*≤0.05; OR 1.94 CI 1.23 to 3.06, *p*≤0.01), at 2 and 6 months following GP consultation, respectively. Additionally, being non-employed and having higher disability scores at baseline improves the chance of developing a persistent pain and disability condition 6 months following this consultation (Table 5). Discrimination of both models (2 and 6 months) was good, with an AUC of 0.86 and 0.83, respectively.

Regarding the MIC criteria, two months after GP’s consultation, and after adjustment, three independent baseline predictors improve the odds of poor outcome, regarding disability, pain and perception of overall change: High scores on the SBST psychosocial subscale (OR: 1.65, 95% CI 1.13–2.40, for pain; OR: 1.61, 95% CI 1.15–2.24, for disability); a LBP episode of more than 3 months duration (OR: 1.71, 95% CI 1.33–1.88, for pain; OR: 1.76, 95% CI 1.43–1.89, for disability), and high levels of pain intensity at baseline for pain (OR: 1.26, 95% CI 1.09–1.39) (Table 4). The discrimination of the different models was acceptable, with an AUC ranging between 0.72 and 0.73.

At 6-months, and after adjustment to significant baseline variables, participants with a LBP episode of less than 12 weeks reduced their probability of poor outcomes on disability, pain and global perception of change (OR: 0.26 95%CI 0.10 to 0.65, *p*≤ 0.01; OR: 0.34 95%CI 0.14 to 0.81, *p*≤0.05, OR: 0.21 95%CI 0.09 to 0.53, *p*≤ 0.01, respectively). The presence of”maladaptive psychosocial factors” (higher psychosocial sub score), however, increased the odds of poor outcomes for disability, pain and global perception of change (OR 2.06 95%CI 1.40 to 3.04, *p*≤ 0.01; 1.82 95%CI 1.27 to 2.59, *p*≤ 0.01; 1.72 95%CI 1.20 to 2.47, *p*≤0.05, respectively). Besides these factors, being employed reduces the chances of poor outcomes on disability (OR 0.31 95%CI 0.11 to 0.92, *p*≤0.05) (Table 4). The discrimination of the different models was acceptable, with an AUC ranging between 0.73 and 0.78.

## Discussion

This study presents the course of the outcomes for patients consulting primary care for an episode of NSLBP. Additionally, it identifies factors associated with the achievement of poor outcomes. Although data was generated from 7 primary care units of a specific health care center, comparison with data from a Portuguese population-based study and other primary care studies suggests that the participants in this study are similar to the Portuguese population with LBP and patients searching for LBP primary care in other countries [4; 16]. Care seeking for a LBP episode is more common in women, and in individuals with poor general health, and with more disabling or more painful episodes [12,13].

The clinical course of disability, pain and HRQoL were favorable with statistical significant differences during the follow-up period (*p*≤0.05). However no additional significant change has been shown to occur between 2 and 6 months. These results are consistent with previous reports and confirm the common trend of early rapid improvement in symptoms that slow down and reach a plateau 6 months after the start of treatment [6; 32].

This study’s findings indicated that 6-month after GP consultation approximately half of the participants reported RMDQ scores compatible with the established definition of persistent disability (RMDQ ≥ 7). When considering the short-term outcomes, half of the NSLBP patients did not reach the MIC criteria (>30% on NPRS and RMDQ), 38% of the patients reported they felt the same or worse, and 76.4% had a poor HRQoL.

Comparisons of the course of outcomes are difficult since many differences exist in terms of the LBP definition used, sample characteristics, length of follow-up or outcomes criteria. For example, in an inception cohort of acute LBP, the cumulative probability of being pain free or having no disability at 6 weeks, defined as being pain-free, or without disability sustained for a whole month, was 39% and 55%, respectively [17]. By 12 weeks the probability increases to 58% and 73%, respectively [17]. In another large cohort study [15] with 521 acute LBP patients, where the authors used the criteria of “fully recovered”, assessed by a general perceived recovery scale, at 6 months, only 19% reported that they weren't “fully recovered”, nor “much improved” (poor outcomes) and 22% had a RMDQ score of ≥7. In a randomized controlled trial with mixed patient populations of LBP, including acute and chronic LBP participants and using the same MIC criteria used in this study for classifying the achievement of poor outcomes (change of <30% from the baseline RMDQ score), 31% to 44% of the participants reported poor outcomes [16]. Thus, this study’s findings indicate a higher rate of poor outcomes but reasons for this difference are difficult to find.

In this study, poor outcomes were consistently associated with a longer duration of the LBP episode and with the presence of maladaptive psychosocial factors (p≤0.05), after adjusting for patient demographic and clinical characteristics. Odds ratios indicated that patients with an episode of pain of less than 12 weeks have a decrease in their likelihood of achieving short-term poor outcomes that vary from 64% to 83%. Moreover, the probability of poor outcomes increases as the psychosocial score of the SBST-PT increases in a range that varies from 57% to 72%. These results suggest that an early identification of the presence of these factors and the implementation of target evidence base interventions might be crucial to decrease the likelihood of poor outcomes and prevent the development of a persistent and disabling LBP condition. Maladaptive psychosocial factors have previously been shown to be strong predictors of poor outcomes [17,18], as well as predictors of chronicity and future disability [19,20] in acute and chronic LBP cohorts. Addressing these factors in primary care at an early stage, before they become well- established and more difficult to treat, could reduce the risk of developing a persistent disabling LBP condition [16; 51].

### Strengths and limitations

The aims of this study were to describe the current health care practice, to examine the clinical course of the outcomes and to identify prognostic indicators for poor outcomes in NSLBP patients who consulted primary care. It is worth noting that the findings of this study emerged from the analysis of the practice in 7 primary care units of a specific health care center, which may limit the generalizability of these findings.

It is also important to note that this study design does not assess the effectiveness of the current health care practice. Although the characteristics of the current health care practice have been recorded and have shown high order rates of imaging and sickness certificates and the use of medication as the first line of treatment, with a small percentage of patients being referred for physiotherapy, this information was based on the data available in the medical records of the GP’s initial appointment. It is therefore possible that not all participants have followed the recommendations of their GP and have decided to not take the prescribed medication or follow other treatments. Therefore, we cannot make any inferences on whether any particular treatment approaches implemented had an influence on outcome rates. Outcome differences found between time points and improvement/non improvement rates could be attributable to the natural history of the condition, regression to the mean, non-specific or specific aspects of the intervention.

The major strengths of this study are the pragmatic nature of this observational study, the minimal loss to follow-up, the use of validated outcome measures, and the low risk of over-fitting of the prediction models.

## Conclusions

This study found that 6-months after consulting primary care for an NSLBP episode approximately half of the participants reported poor outcomes. Furthermore, no additional significant change has been shown to occur between 2 and 6 months, suggesting that any improvement occurs in the first 8 weeks after a LBP onset. Thereafter, the effective management of LBP patients at the early stage of an LBP onset seems to be crucial for the prevention of the development of a persistent disabling back pain condition.

In this study, poor outcomes were consistently associated with a longer duration of the LBP episode and with the presence of maladaptive psychosocial factors. Thus, the early identification of the presence of these factors and the implementation of target evidence base interventions might be crucial to decrease the likelihood of poor outcomes and prevent the development of a persistent and disabling LBP condition.

## Supporting information

S1 File (XLSX)

## List of abbreviations

NLBP: Non-specific low back pain
HRQoL: Health-related quality of life
GP: General Practitioners
CI: confidence intervals
AOR: adjusted odds ratios
LBP: Low back pain
GBD: Global Burden of Disease
STROBE: STrengthening the Reporting of OBservational studies in Epidemiology
RA: research assistant
NPRS: Numeric Pain Rating scale
SBST: Start back screening tool
RMDQ: Roland Morris disability questionnaire
EQ-5D-3L: EuroQol 5-dimension 3-level
GPES: Global Perceived Effect Scale
ICC: intraclass correlation coefficients
MIC: minimal important change
ORs: Odds ratios
AUC: area under the receiver operating characteristic curve
SD: Standard deviation
NSAIDs: Nonsteroidal anti-inflammatory drugs

## References

[1] HartvigsenJ, HancockMJ, KongstedA, LouwQ, FerreiraML, GenevayS, et al What low back pain is and why we need to pay attention. Lancet. 2018;391(10137): 2356–67. 10.1016/S0140-6736(18)30480-X 29573870

[2] Global Burden of Disease, Injury Incidence, Prevalence Collaborators. Global, regional, and national incidence, prevalence, and years lived with disability for 310 diseases and injuries, 1990–2015: a systematic analysis for the Global Burden of Disease Study 2015. Lancet 2016; 388: 1545–602. 10.1016/S0140-6736(16)31678-6 27733282PMC5055577

[3] Global Burden of Disease 2015 DALYs and HALE Collaborators. Global, regional, and national disability-adjusted life-years (DALYs) for 315 diseases and injuries and healthy life expectancy (HALE), 1990–2015: a systematic analysis for the Global Burden of Disease Study 2015. Lancet 2016; 388: 1603–58. 10.1016/S0140-6736(16)31460-X 27733283PMC5388857

[4] BrancoJ, RodriguesAM, GouveiaN, et al (2015). Prevalence of rheumatic and musculoskeletal diseases and their impact on health related quality of life, physical function and mental health in Portugal: results from EpiReumaPt–a national health survey. RMD Open 2016; 2: e000166 10.1136/rmdopen-2015-000166 26848402PMC4731842

[5] da C Menezes CostaL., MaherC. G., HancockM. J., McAuleyJ. H., HerbertR. D., & CostaL. O. P. (2012). The prognosis of acute and persistent low-back pain: a meta-analysis. *CMAJ*, 184(11), E613–24. 10.1503/cmaj.111271 22586331PMC3414626

[6] da CostaLMC, MaherCG, McAuleyJH, et al Prognosis for patients with chronic low back pain: inception cohort study. BMJ 2009; 339: b3829 10.1136/bmj.b3829 19808766PMC2758336

[7] DagenaisS, CaroJ, HaldemanS. A systematic review of low back pain cost of illness studies in the United States and internationally. Spine J 2008; 8: 8–20. 10.1016/j.spinee.2007.10.005 18164449

[8] BalaguéF., MannionA. F., PelliséF., & CedraschiC. (2012). Non-specific low back pain. *Lancet*, 379 (9814), 482–91. 10.1016/S0140-6736(11)60610-7 21982256

[9] JordanKP, KadamUT, HaywardR, PorcheretM, YoungC, CroftP. Annual consultation prevalence of regional musculoskeletal problems in primary care: an observational study. BMC Musculoskelet Disord 2010; 11: 144 10.1186/1471-2474-11-144 20598124PMC2903510

[10] AzevedoL. F., Costa-PereiraA., MendonçaL., DiasC. C., & Castro-LopesJ. M. (2012). Epidemiology of chronic pain: a population-based nationwide study on its prevalence, characteristics and associated disability in Portugal. *The Journal of Pain*, 13(8), 773–83. 10.1016/j.jpain.2012.05.012 22858343

[11] GouveiaN., RodriguesA., EusébioM., RamiroS., MachadoP., CanhãoH., et al (2016). Prevalence and social burden of active chronic low back pain in the adult Portuguese population: results from a national survey. *Rheumatology International*, 36(2), 183–97. 10.1007/s00296-015-3398-7 26661091

[12] FerreiraML, MachadoG, LatimerJ, MaherC, FerreiraPH, SmeetsRJ. Factors defining care-seeking in low back pain—a meta-analysis of population based surveys. Eur J Pain 2010; 14: 747.e1–7 10.1016/j.ejpain.2009.11.005 20036168

[13] MaherC, UnderwoodM, BuchbinderR. Non-specific low back pain. Lancet 2017;389: 736–47. 10.1016/S0140-6736(16)30970-9 27745712

[14] ChouR, ShekelleP. Will this patient develop persistent disabling low back pain? JAMA. 2010; 303: 1295–1302. 10.1001/jama.2010.344 20371789

[15] MehlingWE., Gopisetty, V., Bartmess-LeVasseur, E., Acree, M., Pressman, A., Goldberg, H., et al The Prognosis of Acute Low Back Pain in Primary Care in the U.S. A 2-Year Prospective Cohort Study. Spine (Phila Pa 1976). 2012 4 15; 37(8): 678–684. 10.1097/BRS.0b013e318230ab20 PMC333577322504516

[16] HillJC, WhitehurstDGT, LewisM, et al Comparison of stratified primary care management for low back pain with current best practice (STarT Back): a randomised controlled trial. Lancet 2011; 378:1560–71. 10.1016/S0140-6736(11)60937-9 21963002PMC3208163

[17] HenschkeN, MaherCG, RefshaugeKM, et al Prognosis in patients with recent onset low back pain in Australian primary care: inception cohort study. BMJ 2008;337:a171 10.1136/bmj.a171.10.1136/bmj.a171PMC248388418614473

[18] GeorgeSZ, BeneciukJM. Psychological predictors of recovery from low back pain: a prospective study. BMC Musculoskeletal Disorders. 2015; 16: 49 10.1186/s12891-015-0509-2 25849159PMC4357055

[19] FosterNE, BishopA, ThomasE, MainC, HorneR, WeinmanJ, et al: Illness perceptions of low back pain patients in primary care: what are they, do they change and are they associated with outcome? Pain 2008, 136:177–187. 10.1016/j.pain.2007.12.007 18313853

[20] GrotleM, FosterNE, DunnKM, CroftP: Are prognostic indicators for poor outcome different for acute and chronic low back pain consulters in primary care? Pain 2010, 151:790–797. 10.1016/j.pain.2010.09.014 20932646PMC3398128

[21] ThomasE, SilmanAJ, CroftPR, PapageorgiouAC, JaysonMIV, MacfarlaneGJ. Predicting who develops chronic low back pain in primary care: a prospective study. BMJ 1999;318:1662–7. 10.1136/bmj.318.7199.1662 10373170PMC28145

[22] Schiottz-ChristensenB, NielsenGL, HansenVK, SchodtT, SorensenHT, OlesenF. Long-term prognosis of acute low back pain in patients seen in general practice: a 1-year prospective follow-up study. Fam Pract 1999;16:223–32. 10.1093/fampra/16.3.223 10439974

[23] CampbellP, FosterNadine E., ThomasElaine, and DunnKate M. Prognostic Indicators of Low Back Pain in Primary Care: Five-Year Prospective Study. J Pain. Aug 2013; 14(8): 873–883.10.1016/j.jpain.2013.03.013PMC373900523791041

[24] FosterNE, ThomasE, BishopA, DunnKM, MainCJ. Distinctiveness of psychological obstacles to recovery in low back pain patients in primary care. Pain 2010; 148:398–406. 10.1016/j.pain.2009.11.002 20022697PMC2831173

[25] RamondA, BoutonC, RichardI, RoquelaureY, BaufretonC, LegrandE, et al Psychosocial risk factors for chronic low back pain in primary care—a systematic review. Fam Pract. 2011; 28(1):12–21. 10.1093/fampra/cmq072 20833704

[26] Direção-Geral da Saúde, Institute for Health Metrics and Evaluation. Portugal: The Nation’s Health 1990–2016: An overview of the Global Burden of Disease Study 2016 Results. Seattle, WA: IHME, 2018.

[27] von ElmE, AltmanDG, EggerM, PocockSJ, GøtzschePC, VandenbrouckeJP; STROBE Initiative. The Strengthening the Reporting of Observational Studies in Epidemiology (STROBE)statement: guidelines for reporting observational studies. J Clin Epidemiol. 2008 4;61(4):344–9. 10.1016/j.jclinepi.2007.11.008 .18313558

[28] VandenbrouckeJP, von ElmE, AltmanDG, GøtzschePC, MulrowCD, PocockSJ,et al; STROBE Initiative. Strengthening the Reporting of Observational Studies in Epidemiology (STROBE):explanation and elaboration. Epidemiology. 2007 11;18(6):805–35. 10.1097/EDE.0b013e3181577511 18049195

[29] HoyDG, MarchL, BrooksP, et al Measuring the global burden of low back pain. *Best Pract Res Clin Rheumatol* 2010;24:155–65. 10.1016/j.berh.2009.11.002 20227638

[30] DionneCE, DunnKM, CroftPR, NachemsonAL, BuchbinderR, WalkerBF, et al A consensus approach toward the standardization of back pain definitions for use in prevalence studies. Spine (Phila Pa 1976). 2008; 33: 95–103.1816575410.1097/BRS.0b013e31815e7f94

[31] AiraksinenO, BroxJI, CedraschiC, HildebrandtJ, Klaber-MoffettJ, KovacsF, et al Chapter 4. European guidelines for the management of chronic nonspecific low back pain. Eur Spine J 2006; 15 Suppl 2:S192–300. 10.1007/s00586-006-1072-1 16550448PMC3454542

[32] ArtusM, van der WindtD, JordanKP, CroftPR. The clinical course of low back pain: a meta-analysis comparing outcomes in randomised clinical trials (RCTs) and observational studies. BMC Musculoskelet Disord. 2014;15:68 10.1186/1471-2474-15-68 24607083PMC4007531

[33] MoonsKG, RoystonP, VergouweY, GrobbeeDE, AltmanDG: Prognosis and prognostic research: what, why, and how? BMJ 2009, 338:b375 10.1136/bmj.b375 19237405

[34] HillJC, DunnKM, LewisM, MullisR, MainCJ, FosterNE, et al A primary care back pain screening tool: Identifying patient subgroups for initial treatment. Arthritis Rheum. 2008; 59: 632–41. 10.1002/art.23563 18438893

[35] RolandM, MorrisR. A study of the natural history of back pain. Part I: development of a reliable and sensitive measure of disability in low-back pain. Spine (Phila Pa 1976). 1983;8(2):141–4.622248610.1097/00007632-198303000-00004

[36] GrotleM, BroxJI, VollestadNK. Cross-cultural adaptation of the Norwegian versions of the Roland-Morris Disability Questionnaire and the Oswestry Disability Index. J Rehabil Med 2003; 35:241–7. 10.1080/16501970306094 14582557

[37] MonteiroJ, FaíscaL, NunesO, et al Questionário de Incapacidade de Roland Morris: Adaptação e Validação para os Doentes de Língua Portuguesa com Lombalgia. Acta Med Port 2010; 23:761–766. 21144314

[38] JensenMP, TurnerJA, RomanoJM. What is the maximum number of levels needed in pain intensity measurement? Pain 1994;58:387–92. 10.1016/0304-3959(94)90133-3 7838588

[39] FarrarJ. T., YoungJ. P., LaMoreauxL., WerthJ. L., & PooleR. M. (2001). Clinical importance of changes in chronic pain intensity measured on an 11-point numerical pain rating scale. *Pain*, 94(2), 149–158. 10.1016/s0304-3959(01)00349-9 11690728

[40] ChildsJ. D., PivaS. R., & FritzJ. M. (2005). Responsiveness of the numeric pain rating scale in patients with low back pain. *Spine*, 30(11), 1331–1334. 10.1097/01.brs.0000164099.92112.29 15928561

[41] FerreiraLN, FerreiraPL, PereiraLN. Contributos para a Validação da Versão Portuguesa do EQ-5D. Acta Med Port 2013 Nov-Dec;26(6):664–675.24388252

[42] GroupEuroqol. EQ-5D a measure of health-related quality of life developed by the EuroQol group: user guide. 7th ed Rotterdam: EuroQol Group; 2000.

[43] FerreiraLN, FerreiraPL, PereiraLN et al (2014) The valuation of the EQ-5D in Portugal. Qual Life Res 23(2):413–423. 10.1007/s11136-013-0448-z 23748906

[44] KamperSJ, MaherCG, MackayG. Global Rating of Change Scales: A Review of Strengths and Weaknesses and Considerations for Design. J Man Manip Ther. 2009;17(3):163–70; 10.1179/jmt.2009.17.3.163 20046623PMC2762832

[45] CostaLOP, MaherCG, LatimerJ, FerreiraPH, FerreiraML, 47., PozziGC, et al Clinimetric testing of three self-report outcome measures for low back pain patients in Brazil: Which one is the best? Spine (Phila Pa 1976). 2008;33(22):2459–63.1892332410.1097/BRS.0b013e3181849dbe

[46] FreitasP, PiresD, NunesC, CruzEB (2019) Cross-cultural adaptation and psychometric properties of the European Portuguese version of the Global Perceived Effect Scale in patients with chronic low back pain. Disabil Rehabil. 2019 8 6:1–7. 10.1080/09638288.2019.1648568 31382797

[47] OsteloRW, DeyoRA, StratfordP, WaddellG, CroftP, Von KorffM, et al Interpreting change scores for pain and functional status in low back pain: towards international consensus regarding minimal important change. Spine (Phila Pa 1976). 2008 1 1;33(1):90–4. 10.1097/BRS.0b013e31815e3a10 18165753

[48] Bonferroni, C. E., Teoria statistica delle classi e calcolo delle probabilità, Pubblicazioni del Instituto Superiore di Scienze Economiche e Commerciali di Firenze 193.

[49] FreedmanDA. A note on screening regression equations. Am Stat. 1983;37: 152–155.

[50] HosmerD.W. and LemeshowS. (2000) Applied logistic regression. 2nd Edition, John Wiley & Sons, Inc, New York 10.1002/0471722146

[51] FosterN. Barriers and progress in the treatment of low back pain. BMC Medicine 2011, 9:108 10.1186/1741-7015-9-108 21943396PMC3192671

